The article "Suberoylanilide Hydroxamic Acid, an Inhibitor of Histone Deacetylase, Enhances Radiosensitivity and Suppresses Lung Metastasis in Breast Cancer In Vitro and In Vivo" was published in 2013. Journal: PLoS One.

# Suberoylanilide Hydroxamic Acid, an Inhibitor of Histone Deacetylase, Enhances Radiosensitivity and Suppresses Lung Metastasis in Breast Cancer *In Vitro* and *In Vivo*

**DOI:** 10.1371/journal.pone.0076340

**Published:** 2013-10-10

**Authors:** Hui-Wen Chiu, Ya-Ling Yeh, Yi-Ching Wang, Wei-Jan Huang, Yi-An Chen, Yi-Shiou Chiou, Sheng-Yow Ho, Pinpin Lin, Ying-Jan Wang

**Affiliations:** 1 Department of Environmental and Occupational Health, National Cheng Kung University, Medical College, Tainan, Taiwan; 2 Department of Pharmacology, National Cheng Kung University, Tainan, Taiwan; 3 Graduate Institute of Pharmacognosy, Taipei Medical University, Taipei, Taiwan; 4 Department of Seafood Science, National Kaohsiung Marine University, Kaohsiung, Taiwan; 5 Department of Radiation Oncology, Chi Mei Medical Center, Liouying, Tainan, Taiwan; 6 Division of Environmental Health and Occupational Medicine, National Health Research Institutes, Zhunan, Taiwan; Florida International University, United States of America

## Abstract

Triple-negative breast cancer (TNBC), defined by the absence of an estrogen receptor, progesterone receptor, and human epidermal growth factor receptor 2 expression, is associated with an early recurrence of disease and poor outcome. Furthermore, the majority of deaths in breast cancer patients are from metastases instead of from primary tumors. In this study, MCF-7 (an estrogen receptor-positive human breast cancer cell line), MDA-MB-231 (a human TNBC cell line) and 4T1 (a mouse TNBC cell line) were used to investigate the anti-cancer effects of ionizing radiation (IR) combined with suberoylanilide hydroxamic acid (SAHA, an inhibitor of histone deacetylase (HDAC)) and to determine the underlying mechanisms of these effects *in vitro* and *in vivo*. We also evaluated the ability of SAHA to inhibit the metastasis of 4T1 cells. We found that IR combined with SAHA showed increased therapeutic efficacy when compared with either treatment alone in MCF-7, MDA-MB-231 and 4T1 cells. Moreover, the combined treatment enhanced DNA damage through the inhibition of DNA repair proteins. The combined treatment was induced primarily through autophagy and ER stress. In an orthotopic breast cancer mouse model, the combination treatment showed a greater inhibition of tumor growth. In addition, SAHA inhibited the migration and invasion abilities of 4T1 cells and inhibited breast cancer cell migration by inhibiting the activity of MMP-9. In an *in vivo* experimental metastasis mouse model, SAHA significantly inhibited lung metastasis. SAHA not only enhances radiosensitivity but also suppresses lung metastasis in breast cancer. These novel findings suggest that SAHA alone or combined with IR could serve as a potential therapeutic strategy for breast cancer.

The article "Suberoylanilide Hydroxamic Acid, an Inhibitor of Histone Deacetylase, Enhances Radiosensitivity and Suppresses Lung Metastasis in Breast Cancer In Vitro and In Vivo" was published in 2013. Journal: PLoS One.

## Introduction

Histone acetylation, controlled by histone acetylases and histone deacetylases (HDACs), modifies nucleosome and chromatin structures and regulates gene expression [1], [2]. HDACs are overexpressed in colon, breast, prostate and other cancers, making HDACs an attractive anticancer target [3]–[5]. HDACs have been divided into four classes: class I, class IIa, class IIb, class III and class IV [3]. Previous studies have demonstrated that HDAC inhibitors reverse the aberrant epigenetic changes associated with various cancers and thus are currently being investigated as possible therapeutics [2]. HDAC inhibitors have been shown to induce tumor cell differentiation, apoptosis, and/or growth arrest in several *in vitro* and *in vivo* experimental models [2]. One of these HDAC inhibitors, suberoylanilide hydroxamic acid (SAHA), has been Food and Drug Administration approved for patients with cutaneous T-cell lymphoma who have failed prior therapies [6]. Data from clinical trials show that SAHA is well tolerated and has limited toxicity which is rapidly reversible upon discontinuation of the drug [7], [8]. SAHA has been shown to inhibit HDAC activity and enhance radiosensitivity in multiple cell lines [9]–[11]. However, there is limited data investigating SAHA in the metastatic setting. Recently, it was reported that SAHA inhibits brain metastatic colonization in a model of triple-negative breast cancer and induces DNA double-strand breaks (DSBs) [12]. Previous studies have demonstrated that the expression of matrix metalloproteinase-9 (MMP-9) has been associated with a high potential of metastasis in several human carcinomas including breast cancer [13]. Our group has shown that HTPB, a novel HDAC inhibitor, inhibits lung cancer cell migration via reduced activities of MMPs, RhoA, and focal adhesion complex [14].

HDAC inhibitors can induce cell-cycle arrest, promote differentiation, stimulate ROS generation, inhibit tumor angiogenesis and induce apoptosis [3]. More recently, HDAC inhibition has been shown to induce autophagy [15], [16]. Autophagy is a catabolic process by which cytosolic material is targeted for lysosomal degradation by means of double-membrane-bound cytosolic vesicles, termed autophagosomes [17]. During autophagy, free cytosolic LC3 (termed LC3-I) becomes conjugated to phosphatidylethanolamide (termed LC3-II). LC3-II is then incorporated into the growing autophagosome structure that, upon maturation, fuses with the lysosome compartment, leading to the degradation of the autophagosome contents [18]. Autophagic cell death is another important physiological cell death process. SAHA has been reported to induce autophagy, which may contribute to its anticancer activity [16]. The excessive number of cells undergoing “self-eating” through autophagy during chemotherapy may trigger cell death by an as yet unknown mechanism.

The article "Suberoylanilide Hydroxamic Acid, an Inhibitor of Histone Deacetylase, Enhances Radiosensitivity and Suppresses Lung Metastasis in Breast Cancer In Vitro and In Vivo" was published in 2013. Journal: PLoS One.

Increasing evidence in the literature shows that DNA damage induces autophagy, but the role of autophagy in the DNA damage response is still unclear [19]–[21]. Ionizing radiation (IR) leads to cell death through the induction of DSBs. Cells have developed mechanisms to repair such DSBs through two major pathways: non-homologous end joining (NHEJ) and homologous recombination (HR). HDACs influence the DNA damage response through the acetylation of key DNA repair and checkpoint proteins [22]. It has been demonstrated that HDAC inhibitors inhibit DNA repair by downregulation or inhibition of the activity of DNA repair proteins, including the components of the NHEJ and HR pathways in cancer cells [23], [24]. Therefore, HDAC inhibitors showed promise as radiosensitizers when administered in combination with radiotherapy [25]. In addition, recent evidence has shown that one of the mechanisms whereby IR activates endoplasmic reticulum (ER) stress is by the induction of DNA damage [26]. The ER plays an important role as a sensor for cellular stress to detect the changes in cell homeostasis and responds to different signaling pathways [27]. There are three main pathways that mediate ER stress: the inositol-requiring enzyme 1 (IRE1) pathway; the PKR-like ER-resistant kinase (PERK) pathway; and the activating transcription factor 6 (ATF6) pathway [28]. Many chemotherapeutic agents and IR-induced ER stress can lead to apoptosis or autophagy in cancer cells [29]–[31]. A recent study indicated that HDAC inhibitors induced autophagy through the downregulation of Akt/mTOR signaling and the induction of the ER stress response in hepatocellular carcinoma cells [32]. Although autophagy has been associated with ER stress, the detailed molecular mechanism behind the activation of autophagy under ER stress is still not fully elucidated.

Triple-negative breast cancer (TNBC) is characterized by a lack of receptor expression of the estrogen receptor (ER), progesterone receptor (PR) and human epidermal growth factor receptor 2 (HER2) [33]. TNBC exhibits characteristics quite distinct from other types of breast cancers, presenting as an aggressive disease that recurs and metastasizes more often than other types of breast cancers [34]. In the present study, MCF-7 (an estrogen receptor-positive human breast cancer cell line), MDA-MB-231 (a human TNBC cell line) and 4T1 (a mouse TNBC cell line) were used to investigate the anti-cancer effects of IR combined with SAHA. Furthermore, we have tested the inhibitory effect of IR combined with SAHA on a 4T1 murine orthotopic breast cancer model. The types of cell death induced by IR when combined with SAHA were examined. We also evaluated the anti-metastatic effects of SAHA in 4T1 cells.

The article "Suberoylanilide Hydroxamic Acid, an Inhibitor of Histone Deacetylase, Enhances Radiosensitivity and Suppresses Lung Metastasis in Breast Cancer In Vitro and In Vivo" was published in 2013. Journal: PLoS One.

## Materials and Methods

### Cell Culture

The mouse breast cancer cell line 4T1 (ATCC CRL-2539) and human breast cancer cell lines MCF-7 (ATCC HTB-22) and MDA-MB-231 (ATCC HTB-26) were obtained from the American Type Culture Collection (ATCC). The luciferase-expressing murine breast cancer cell line, 4T1-Luc, was obtained from Dr. M.L. Kuo (Institute of Toxicology, National Taiwan University, Taipei, Taiwan) [35]. The cells were cultured in Dulbecco’s modified essential medium (DMEM) (Gibco BRL, Grand Island, NY) supplemented with antibiotics containing 100 U/ml penicillin, 100 µg/ml streptomycin (Gibco BRL, Grand Island, NY) and 10% fetal bovine serum (HyClone, South Logan, UT, USA).The cells were incubated in a humidified atmosphere containing 5% CO_2_ at 37°C. Exponentially growing cells were detached using 0.05% trypsin-EDTA (Gibco BRL, Grand Island, NY) in DMEM medium.

### Irradiation Treatment and Cell Viability Assay

IR was performed with 6 MV X-rays using a linear accelerator (Digital M Mevatron Accelerator, Siemens Medical Systems, CA, USA) at a dose rate of 5 Gy/min. An additional 2 cm of a tissue-equivalent bolus was placed on the top of the plastic tissue-culture flasks to ensure electronic equilibrium, and 10 cm of tissue-equivalent material was placed under the flasks to obtain full backscatter. After IR treatment, cells were treated with SAHA immediately. The treated cells were centrifuged and were then resuspended in 0.1 ml PBS. Each cell suspension (0.02 ml) was mixed with 0.02 ml trypan blue solution (0.2% in PBS). After 1 or 2 min, each solution was placed on a hemocytometer, and the blue-stained cells were counted as nonviable.

### Clonogenic Assay

The cells were irradiated using the dosages of 2, 4 or 6 Gy. SAHA was added to the cells at concentrations of 3 or 5 µM. The cells were trypsinized and counted. Known numbers of cells were subsequently replated in 6-cm culture dishes and returned to the incubator to allow for colony development. After 10 days, colonies (containing ≥50 cells) were stained with 0.5% crystal violet solution for 30 min. The plating efficiency (PE) is the ratio of the number of colonies to the number of cells seeded in the nonirradiated group. Calculation of survival fractions (SFs) was performed using the equation: SF = colonies counted/(cells seeded×PE), using the individual PE. In the survival curve analysis, the one of major parameters for intrinsic radiation sensitivity is the D_0_ value, which is determined from the straight portion of the radiation dose survival curve as the dose required to reduce the fraction of surviving cells to 37% [36].

The article "Suberoylanilide Hydroxamic Acid, an Inhibitor of Histone Deacetylase, Enhances Radiosensitivity and Suppresses Lung Metastasis in Breast Cancer In Vitro and In Vivo" was published in 2013. Journal: PLoS One.

### Comet Assay

To detect DNA damage in individual cells, we adopted a comet assay. Briefly, cells (2×10^4^) were collected after the treatments and resuspended in 0.2 ml PBS containing 0.5% low-melting-point agarose. Eighty-five microliters of the mixture was applied to slides, which were then submerged in cold lysis solution (2.5 M NaCl, 0.1 M EDTA, 10 mM Tris, 1% Triton X-100 (pH 10)). Electrophoresis was performed at 300 mA and 25 V for 20 min. After electrophoresis, the slides were neutralized with 0.4 M cold Tris-HCl buffer (pH 7.5) and then stained using ethidium bromide. Comets were visualized using a fluorescence microscope (Olympus, Japan). DNA damage was assessed in 100 cells where tail moment (tail length multiplied by the fraction of DNA in the tail) was quantified using Image-Pro Plus (Media Cybernetics Inc.).

### Staining of ER

Cells were treated with various treatments for 24 hrs. ER-Tracker Blue-White DPX (Molecular Probes, Eugene, OR) probe was added to the cells and incubated for 30 min under the same growth conditions. The loading solution was removed, and cells were then washed with PBS. Microscopic images were collected using the fluorescence microscope.

### Determination of Early Apoptosis

Apoptosis was assessed by quantifying the translocation of phosphatidylserine to the cell surface, detected with an Annexin V apoptosis detection kit (Calbiochem, San Diego, CA, USA), according to our previous report [37].

### Supravital Cell Staining with Acridine Orange for Detection of Autophagy

Cell staining with acridine orange (Sigma Chemical Co.) was performed according to published procedures [37].

### Immunofluorescence Microscopy

Cells were fixed in 4% paraformaldehyde and blocked with 1% BSA for 30 min. This was followed by incubation in specific antibodies against LC3 (MBL, Japan) for 1 hr. After washing, cells were labeled with a DyLight™ 488-conjugated affinipure goat anti-rabbit IgG (Jackson ImmunoResearch Laboratories, PA, USA) for 1 hr. Finally, cells were washed in PBS, coverslipped, and examined with a fluorescence microscope. To quantify LC3-positive cells, a minimum of 50 cells per sample was counted, and the number of LC3 aggregates was enumerated. Cells were scored as positive if they had more than ten LC3 puncta, and the data were presented as a percentage of the total number of LC3-positive cells.

### Electron Microscopy

Cells were fixed using a solution containing 2.5% glutaraldehyde and 2% paraformaldehyde in 0.1 M cacodylate buffer, pH 7.3, for 1 hr. After fixation, the samples were postfixed in 1% OsO_4_ in the same buffer for 30 min. Ultra-thin sections were subsequently observed under a transmission electron microscope (JEOL JEM-1200EX, Japan) at 100 kV.

The article "Suberoylanilide Hydroxamic Acid, an Inhibitor of Histone Deacetylase, Enhances Radiosensitivity and Suppresses Lung Metastasis in Breast Cancer In Vitro and In Vivo" was published in 2013. Journal: PLoS One.

### Western Blot Analysis

Total cellular protein lysates were prepared by harvesting cells in protein extraction buffer for 1 hr at 4°C, as described previously [38]. GAPDH expression was used as the protein loading control. Antibody for detecting anti-GAPDH was obtained from Abcam (Cambridge, MA, USA); anti-acetyl-histone H3 and acetyl-histone H4 antibodies were obtained from Millipore (Bedford, MA, USA); anti-acetyl-tubulin antibody was obtained from Sigma (St. Louis, Missouri, USA); anti-LC3 and anti-eIF2αantibodies were obtained from Abgent (San Diego, CA, USA); anti-MMP-9 antibody was obtained from Cell Signaling Technology (Ipswich, MA, USA), and anti-Beclin 1, anti-IRE1α, anti-phospho-eIF2α, anti-Rad51, anti-DNA-PK and anti-γH2AX antibodies were obtained from Epitomics (Burlingame, CA, USA).

### Wound Healing Assay

The cells were carefully scratched using a plastic pipette tip to draw a linear “wound” in the cell monolayer of each well. Cells were then treated with different concentration of SAHA for 24 hrs. Under the microscope, the number of cells that migrated into the cell-free zone, based on the zero line of the linear “wound,” was evaluated. Three independent experiments were photographed and quantified under a microscope.

### Transwell Migration Assay and Matrigel Invasion Assay

The migratory ability of 4T1 cells was determined using Transwell insert (8 µm pore size) (Millipore Corp., Bedford, MA). The upper compartment contained 3×10^4^ cells in 100 µl of serum-free medium with or without SAHA; the lower compartment contained culture medium with 10% FBS. After 24 hrs, nonmigrating cells were scraped from the upper surface of the membrane with a cotton swab, and the cells remaining on the bottom surface were counted after staining with 0.5% crystal violet. Evaluation of completed transmigration was performed under the microscope, and random fields were scanned (three fields per filter) for the presence of cells at the lower membrane side only. Similar to the Transwell migration assay, the Matrigel invasion assay was also determined by using a Transwell insert (8-µm pore, BD Biosciences, California, USA), that was precoated with 20-µg Matrigel (BD Bioscience) in DMEM medium. The other experimental procedures were the same as for the Transwell migration assay.

### Gelatin Zymography Assay

Conditioned medium was collected from cells treated with SAHA for 24 hrs, and analyzed by gelatin zymography in 0.1% gelatin-8% acrylamide gels. After electrophoresis, gels were washed with 2.5% Triton X-100 to remove SDS and renatured in MMP-9 in the gel. Then, the gels were incubated in the developing buffer overnight to induce gelatin lysis by renatured MMP-9. The gel was then stained with 0.25% Coomassie blue for 30 min. Proteolytic activity was identified as the presence of clear bands in the gel.

The article "Suberoylanilide Hydroxamic Acid, an Inhibitor of Histone Deacetylase, Enhances Radiosensitivity and Suppresses Lung Metastasis in Breast Cancer In Vitro and In Vivo" was published in 2013. Journal: PLoS One.

### Ethics Statement

All experiments on mice were performed according to the guidelines of our institute (the Guide for Care and Use of Laboratory Animals, National Cheng Kung University Medical College). The animal use protocol listed below has been reviewed and approved by the Institutional Animal Care and Use Committee of National Cheng Kung University, Taiwan (Approval No: 101107). All surgical procedure was performed under isoflurane anesthesia (Minrad Inc, PA, USA) and all efforts were made to reduce unnecessary pain.

### Orthotopic Breast Cancer Model

Five- to six week-old female Balb/c mice were acquired from the National Laboratory Animal Center (Taiwan). The animals were housed five per cage at 24±2°C and 50% ±10% relative humidity and subjected to a 12-h light/12-h dark cycle. The animals were acclimatized for 1 week prior to the start of experiments and fed with a Purina chow diet and water ad libitum. 4T1-luc cells (5×10^4^ cells in 0.2 ml of PBS) were injected into the lactiferous ducts of the 4th mammary fat pads of the female Balb/c mice. Seven days of postinoculation, the mice were randomized into five groups (5 mice per group): (1) normal: untreatment. (2) control (DMSO): mice were injected (intraperitoneally, i.p.) with DMSO. (3) SAHA group: mice were injected i.p. with 25 mg/kg SAHA three times per week for three weeks. (4) IR group: mice were treated with a single dose of 4 Gy IR. (5) SAHA+IR: mice were treated with a combination of treatments with 25 mg/kg SAHA three times per week and a single dose of 4 Gy IR in the beginning of first week. About the procedure of IR treatment, mice were anesthetized and treated with 6 MV X-rays using a linear accelerator at a dose rate of 5 Gy/min in 4th mammary fat pads. After IR treatment, the combination of SAHA and IR group was treated with SAHA immediately. Bioluminescence imaging was conducted using an IVIS 200 imaging system coupled to a data acquisition computer running Living Image Software (XENOGEN). Before imaging, mice were anesthetized with isoflurane and injected i.p with 150 mg/kg body weight endotoxin-free luciferase substrate (VivoGlo™, Promega). Mouse body weights were measured once per week and were used as an indicator of the systemic toxicity of the treatment. There were no deaths in all groups during the experimental period. Mice were sacrificed via CO_2_ exposure. After sacrificed, the tumor tissues were formalin fixed and paraffin embedded for immunohistochemistry.

The article "Suberoylanilide Hydroxamic Acid, an Inhibitor of Histone Deacetylase, Enhances Radiosensitivity and Suppresses Lung Metastasis in Breast Cancer In Vitro and In Vivo" was published in 2013. Journal: PLoS One.

### *In vivo* Experimental Metastasis Assay

Five- to six week-old female Balb/c mice were acquired from the National Laboratory Animal Center (Taiwan). 4T1-luc cells were intravenously injected into the tail-vein of Balb/c mice. The mice were randomized into three groups (5 mice per group): (1) normal: untreatment. (2) control (DMSO): mice were injected i.p. with DMSO. (3) SAHA group: mice were injected i.p. with 25 mg/kg SAHA three times per week for three weeks. Mouse body weights were measured once per week and were used as an indicator of systemic toxicity of the treatment. Before sacrifice, mice were anesthetized and injected with 150 mg/kg body weight endotoxin-free luciferase substrate (VivoGlo™, Promega). Then, tumor volumes were monitored using the IVIS 200 imaging system (XENOGEN). There were no deaths in all groups during the experimental period. Mice were sacrificed via CO_2_ exposure. After sacrifice, the metastasized tumor nodules in the lung tissue were dissected and H&E-stained for further confirmation.

### Immunohistochemical (IHC) Staining Analysis

Paraffin-embedded tissue sections (4 µm) were dried, deparaffinized, and rehydrated. Following microwave pretreatment in citrate buffer (pH 6.0; for antigen retrieval), the slides were immersed in 3% hydrogen peroxide for 20 min to block the activity of endogenous peroxidase. After extensive washing with PBS, the slides were incubated overnight at 4°C with the anti-LC3 (MBL, Japan) or anti-γH2AX (Epitomics, USA) antibodies. The sections were then incubated with a secondary antibody for 1 hr at room temperature, and the slides were developed using the STARR TREK Universal HRP detection kit (Biocare Medical, Concord, CA). Finally, the slides were counterstained using hematoxylin. Each slide was imaged at low magnification (×100).

### Biochemistry Tests

Whole blood samples from treated mice were collected by intracardiac puncture and centrifuged at 2000×g for 20 min to separate the serum. Biochemistry evaluation included glutamate oxaloacetate transaminase (GOT) activity, glutamate pyruvate transaminase (GPT) activity, albumin levels, blood urea nitrogen (BUN) levels and creatinine levels. All experiments and procedures were performed in accordance with the Institutional Care Use Committee guidelines.

### Statistical Analysis

Data are expressed as the mean ± SD. Statistical significance was determined using Student’s t-test for comparison between the means or one-way analysis of variance with post-hoc Dunnett’s test [39]. Differences were considered to be significant when p<0.05.

The article "Suberoylanilide Hydroxamic Acid, an Inhibitor of Histone Deacetylase, Enhances Radiosensitivity and Suppresses Lung Metastasis in Breast Cancer In Vitro and In Vivo" was published in 2013. Journal: PLoS One.

## Results

### Cytotoxic Effects and Survival Curves of SAHA and IR Treated Alone or in Combination on Breast Cancer Cells

The biomarkers of HDAC inhibition are acetylation of histone and non-histone proteins [40]. Exposure to SAHA induced acetylation of histone H3, histone H4 and tubulin in a concentration-dependent manner (Fig. 1A). The viability of the cells was observed at different concentrations (or doses) of SAHA or IR for 24 hrs in MCF-7, MDA-MB-231 and 4T1 cells (Figs. 1B&1C). SAHA or IR alone reduced the viability of cells in a concentration (or dose)-dependent manner. Figure 1D shows the viability of breast cancer cells treated with SAHA or IR treated alone or in combination. Significantly enhanced toxicity in breast cancer cells was found for the combined treatment compared with SAHA or IR treatment alone for 24, 36 and 48 hrs. Furthermore, figures 1E&1F show that the radiation dose–response survival curves for 4T1 cells with increasing doses of SAHA shift downward. Thus, SAHA (3 or 5 µM) treatment increased IR-induced clonogenic cell death in 4T1 cells and significantly reduced the survival fraction in a dose-dependent manner compared to IR alone. D_0_ of IR treatment alone, combined with SAHA (3 µM) and SAHA (5 µM) treatment were 4.03, 3.56 and 3.21, respectively.

**Figure 1:** IR dose–response survival curves and cytotoxic effects resulting from SAHA and/or IR treatment in breast cancer cells. (A) Concentration-dependent effects of SAHA on histone and nonhistone proteins for 24 hrs in 4T1 cells. (B) Concentration-dependent effects of SAHA on the viability of breast cancer cells. Cells were treated with 1, 3, 5 or 7 µM SAHA for 24 hrs. *, *p*<0.05, SAHA versus control. (C) Dose-dependent effects of IR on the viability of breast cancer cells. Cells were treated with 2, 4, 6 or 8 Gy IR for 24 hrs. *, *p*<0.05, IR versus control. (D) Cytotoxic effects in cells treated with IR (4 Gy) and/or SAHA (3 µM). #, *p*<0.05, IR versus combined treatment. *, *p*<0.05, SAHA versus combined treatment. (E) Clonogenic assay in 4T1 cells treated with IR (4 Gy) and/or SAHA (3 µM). (F) The radiation dose-response survival curves of 4T1 cells with or without SAHA. Data are presented as the mean ± standard deviation of three independent experiments.

### Effect of DNA Damage, DNA Repair and ER Stress in 4T1 Cells Treated with SAHA and IR Alone or in Combination

Exposure of cells to IR causes DNA damage, followed by the formation of phosphorylated histone variant H2AX (γH2AX) [41]. Our results showed that the expression level of γH2AX increased significantly at 15 and 30 min after IR compared to controls (Fig. 2A). However, γH2AX decreased in cells treated with IR treatment after 30 min. Furthermore, the expression level of γH2AX was significantly enhanced for the combined treatment compared with SAHA or IR alone (Fig. 2B). SAHA has been found to downregulate DNA repair-related proteins, such as Rad51 and DNA-PK (Fig. 2B). The comet assay is a sensitive tool for the estimation of DNA damage and repair at the cellular level, requiring only a small number of cells [42]. In the comet assay for the 4T1 cells, significantly enhanced DNA damage was found for the combined treatment compared with SAHA and IR alone (Fig. 2C). Our results suggest that SAHA lowers the cell’s capacity to repair IR-induced DNA damage by affecting the DNA repair pathways. In addition, recent evidence shows that one of the mechanisms whereby IR activates ER stress is through the induction of DNA damage [26]. It has been reported that the induction of ER stress by treatment with thapsigargin, an ER Ca^2+^-ATPase inhibitor, increases the fluorescence intensity of ER-Tracker Blue-White DPX, an ER-specific dye [43]. Our results showed that the treatment of cells with SAHA, IR and combined treatment significantly increased the staining intensity of this dye, suggesting a possible induction of ER stress (Fig. 2D). ER stress has been reported to connect autophagy through the PERK/eIF2α and IRE1/TRAF/JNK signaling pathways [44]. We therefore examined whether ER stress signaling was involved in combined treatment-induced autophagy in 4T1 cells (Fig. 2E). Phosphorylation of eIF2α increased in 4T1 cells treated with IR or SAHA alone or in combination. IRE1α expression increased in cells treated with combined IR and SAHA compared with those subjected to individual treatment.

The article "Suberoylanilide Hydroxamic Acid, an Inhibitor of Histone Deacetylase, Enhances Radiosensitivity and Suppresses Lung Metastasis in Breast Cancer In Vitro and In Vivo" was published in 2013. Journal: PLoS One.

**Figure 2:** DNA damage, DNA repair and ER stress induced by IR and/or SAHA in 4T1 cells. (A) Time-dependent effects of IR on the expression of γH2AX. Cells were treated with IR (4 Gy). (B) Western blotting for γH2AX, Rad51 and DNA-PK in 4T1 cells. (C) Comet assay induced by IR and/or SAHA. The tails indicate DNA damage. The effect of SAHA (3 µM) or IR (4 Gy) alone or in combination for 24 hrs on average tail DNA. #, *p*<0.05, IR versus combined treatment. *, *p*<0.05, SAHA versus combined treatment. (D) ER staining enhanced by IR and/or SAHA. Cells were treated with IR (4 Gy) and SAHA (3 µM) for 24 hrs and treated with ER Tracker Blue-White DPX for ER staining. (E) Western blotting for IRE1α, phospho-eIF2α and eIF2 in 4T1 cells. Cells were treated with IR (4 Gy) and SAHA (3 µM) for 24 hrs.

### Measurement of Apoptosis and Autophagy in Breast Cancer Cells Treated with SAHA or IR Alone or in Combination

As shown in Figure 3A, early apoptosis in 4T1 and MDA-MB-231 cells was measured by flow cytometry with the Annexin V apoptosis detection kit. Quantitative results showed that the occurrence of early apoptosis in 4T1 and MDA-MB-231 cells treated with SAHA and/or IR was low. Thus, we further analyzed the occurrence of type II programmed cell death, autophagy, which is characterized by the formation of numerous acidic vesicles that are called acidic vesicular organelles (AVOs) [45]. Microphotographs of AVOs were observed as green and red fluorescence in acridine orange (AO)-stained cells by using a fluorescence microscope (Fig. 3B). AO staining was quantified using flow cytometry (Fig. 3C). A significant increase in AO-positive cells was found for cells receiving the combined treatment as compared to those treated with IR or SAHA alone in 4T1 and MDA-MB-231 cells. Furthermore, to detect the expression of autophagy-related proteins, we performed western blotting with lysates from 4T1 cells that received each of the different treatments (Fig. 3D). The expression levels of LC3-II and Beclin 1 proteins increased with combined treatment. In addition, we applied fluorescence microscopy to determine the percentage of cells with punctate LC3 staining (Fig. 3E). The results showed that combined treatment increased the percentage of LC3 puncta of 4T1 cells. The ultrastructures of the 4T1 cells for each treatment group were observed by EM photomicrography (Fig. 3F). The combined treatment also resulted in a large number of autophagic vacuoles and autolysosomes in the cytoplasm. In addition, no significant chromatin condensation or nuclear pyknosis, which are characteristic of apoptosis, were observed in the treated cells. Next, we used 3-methyladenine (3-MA), an inhibitor of autophagy, to determine whether inhibition of autophagy alters combined treatment-induced cytotoxicity (Fig. 3G). The results indicated that combined treatment with 3-MA revealed a significant decrease of cytotoxicity compared to combined treatment. These results confirm that the combined treatment induced more autophagy than apoptosis in 4T1 cells.

**Figure 3:** Measurement of apoptosis and autophagy in breast cancer cells that received various treatments. (A) Early apoptosis, detected using an Annexin V apoptosis detection kit, was measured using flow cytometry. Cells were treated with IR (4 Gy) and SAHA (3 µM) for 6, 12 or 24 hrs. (B) Microphotograph of AVOs in 4T1 cells. Detection of green and red fluorescence in acridine orange (AO)-stained cells was performed using a fluorescence microscope. Cells were treated with IR (4 Gy) and SAHA (3 µM) for 24 hrs. (C) Quantification of AVOs with AO-stained cells treated with IR (4 Gy) or SAHA (3 µM) alone or in combination using flow cytometry. #, *p*<0.05, IR versus combined treatment. *, *p*<0.05, SAHA versus combined treatment. (D) Western blotting for LC3-I, LC3-II and Beclin 1 in 4T1 cells. Cells were treated with IR (4 Gy) and SAHA (3 µM) for 12 hrs. (E) Immunofluorescence staining of LC3 protein in 4T1 cells treated with IR (4 Gy) and SAHA (3 µM) for 12 hrs. #, *p*<0.05, IR versus combined treatment. *, *p*<0.05, SAHA versus combined treatment. (F) EM microphotographs of 4T1 cells treated with IR (4 Gy) and SAHA (3 µM) for 24 hrs. The *black arrows* point to autophagic vacuoles and autolysosomes. (G) Cytotoxic effects in the absence or presence of 3-MA. Cells were pretreated with 3-MA for 1 hr before combined treatment. *, *p*<0.05, combined treatment versus combined treatment +3-MA. Data are presented as the mean ± standard deviation of three independent experiments.

The article "Suberoylanilide Hydroxamic Acid, an Inhibitor of Histone Deacetylase, Enhances Radiosensitivity and Suppresses Lung Metastasis in Breast Cancer In Vitro and In Vivo" was published in 2013. Journal: PLoS One.

### Tumor Growth in an Orthotopic Breast Cancer Model was Suppressed by IR and SAHA

We examined the therapeutic potential of IR and SAHA either alone or in combination on the growth of orthotopically implanted human breast cells in Balb/c mice. We measured the body weight of the mice on weekly basis. The results of this study demonstrated that none of the treatment regimens produced any loss of body weight, which may serve as a sign of toxicity (Fig. 4A). In addition, treatment with SAHA caused no detectable toxicity as examined by biochemistry examination (Table 1). The IVIS imaging was performed every week after tumor implantation (Figs. 4B&4C). The bioluminescence imaging results showed a gradual increase in tumor volume in the control group in a time-dependent manner. The tumor volume in the combination of SAHA and IR group was significantly lower than in the control group. Next, the LC3 and γH2AX expression patterns in tumors were examined using IHC staining (Fig. 4D). LC3 and γH2AX were increased in tumors from mice treated with the combined treatment compared with SAHA or IR treatment alone.

**Figure 4:** Tumor growth and body weight of the orthotopic breast cancer model mice treated with IR (4 Gy) or SAHA (25 mg/kg×9) alone or in combination. (A) Body weight in Balb/c mice measured once per week. (B) The 4T1-luc cells were injected into mammary fat pads of Balb/c mice, observed for luciferase signals and photographed using IVIS 200. (C) Quantification of the luciferase signals. *, *p*<0.05, versus control. (D) IHC staining of the mouse orthotopic tumor tissues. IHC was used to determine the expression levels of LC3 and γH2AX (×100 objective magnification). The percentage of LC3 and γH2AX-positive cells was determined using HistoQuest software (TissueGnostics).

The article "Suberoylanilide Hydroxamic Acid, an Inhibitor of Histone Deacetylase, Enhances Radiosensitivity and Suppresses Lung Metastasis in Breast Cancer In Vitro and In Vivo" was published in 2013. Journal: PLoS One.

**Table 1:** Biochemistry tests including GOT, GPT, albumin, BUN, and creatinine.

		4T1-Luc cells			
Item/Group	Normal	Control	SAHA	IR	SAHA+IR
**GOT (U/l)**	111±6	122±6	123±9	132±4	130±12
**GPT (U/l)**	34±3	25±2	28±3	28±1	38±2
**Albumin (g/dl)**	1.6±0.0	1.7±0.1	1.6±0.1	1.6±0.1	1.7±0.0
**BUN (mg/dl)**	18.0±1.5	22.4±3.1	16.5±2.0	15.5±1.0	17.3±0.5
**Creatinine (mg/dl)**	0.1±0.0	0.2±0.0	0.1±0.0	0.2±0.1	0.2±0.0

### SAHA Inhibits Migratory and Invasive Abilities of 4T1 Cells

To investigate the effect of SAHA on breast cancer cell motility, doses of SAHA that did not affect cell viability were chosen (Fig. 5A), so that the antimetastatic effects could be further studied unambiguously. The results showed that the noncytotoxic SAHA treatment significantly decreased the cell migration of 4T1 cells for 24 hrs, as measured by wound-healing assay and Trans-well migration assay of 4T1 cells (Figs. 5B&5C). Moreover, in Matrigel invasion assay, SAHA significantly inhibited the invasive ability of 4T1 cells (Fig. 5D). We also assessed the effect of SAHA on MMP-9 activity by gelatin zymography, which is related to the invasive and metastatic properties of cancer cells. As shown in Figure 5E, SAHA dramatically inhibited the proteolytic activity of MMP-9 in a concentration-dependent manner. Furthermore, we analyzed the effect of SAHA on the levels of MMP-9 protein in 4T1 cells and found that the expression levels of MMP-9 protein decreased with SAHA treatment as evidenced by western blot analysis (Fig. 5F). These results suggested that SAHA decreased migration and invasion of breast cancer cells partly through inhibiting the activity of MMP-9 protein.

**Figure 5:** Effects of SAHA on cell viability, migration and invasion of 4T1 cells. (A) Concentration-dependent effects of SAHA on the viability of 4T1 cells. SAHA inhibits 4T1 cell migration in a wound healing assay (B) and Trans-well migration assay (C). (D) The invasive ability of 4T1 cells was determined using a Matrigel invasion assay. MMP-9 enzyme activity was determined using a gelatin zymography assay (E) and western blot analysis (F) of conditioned medium. Cells were treated with SAHA for 24 hrs. Data are presented as the mean ± standard deviation of three independent experiments.

### SAHA Significantly Inhibits Breast Cancer Cell Metastasis *in vivo*

We further examined the therapeutic efficacy of SAHA against tumor metastasis. For this purpose, 4T1-luc cells were injected into Balb/c mice via tail vein to imitate tumor metastasis. As shown in Figure 6A, throughout the experiment there was no noticeable difference in body weight between the mice treated with SAHA and those that were not treated, indicating that the intraperitoneal administration of SAHA did not lead to remarkable toxicity. Furthermore, significantly lower lung weight was observed in mice treated i.p. with SAHA than in control mice (Fig. 6B). Then, tumor volumes were monitored using the IVIS 200 imaging system. The data indicate that SAHA significantly decreases lung metastasis of 4T1-luc cells compared to control (Fig. 6C). After sacrifice, the lung tissues were dissected and H&E-stained for further confirmation. A significant decrease in the number and size of tumors was observed in the lung sections from animals treated with SAHA compared to controls (Fig. 6D). In addition, treatment with SAHA caused no detectable toxicity as examined by biochemistry examination (Table 2). These results suggested that SAHA could inhibit metastasis of 4T1-luc cells *in vivo*.

The article "Suberoylanilide Hydroxamic Acid, an Inhibitor of Histone Deacetylase, Enhances Radiosensitivity and Suppresses Lung Metastasis in Breast Cancer In Vitro and In Vivo" was published in 2013. Journal: PLoS One.

**Figure 6:** SAHA inhibits experimental metastasis in Balb/c mice. (A) Body weight in Balb/c mice measured once per week. (B) Lung weights of mice. *, *p*<0.05, versus control. (C) The 4T1-luc cells were observed for the luciferase signals and photographed using IVIS 200. (D) Histological characteristics of mouse lungs stained with H&E. Tumor metastasis is indicated by arrows.

**Table 2:** Biochemistry tests including GOT, GPT, albumin, BUN, and creatinine.

		4T1-Luc cells	
Item/Group	Normal	Control	SAHA
**GOT (U/l)**	103±19	111±6	114±19
**GPT (U/l)**	36±1	30±4	28±4
**Albumin (g/dl)**	2.0±0.2	1.9±0.1	1.9±0.2
**BUN(mg/dl)**	16.7±1.7	16.3±0.6	15.5±1.0
**Creatinine (mg/dl)**	0.1±0.0	0.2±0.0	0.1±0.0

## Discussion

HDAC inhibitors are currently used in cancer treatment. Additionally, multiple HDAC inhibitors have also been shown to affect radiosensitivity in preclinical models [2], [46]. To investigate the importance of protein acetylation in the DSB repair pathway [47], SAHA treatment in combination with IR has been reported to attenuate both the upregulation of IR-induced Rad50 in melanoma cell lines [10] and the upregulation of DNA-PK protein levels in prostate cancer cells [9]. In terms of HR, SAHA attenuates Rad51 upregulation in melanoma and rhabdomyosarcoma cells after IR [48]. In the present study, we found that SAHA enhanced DNA damage after IR through the inhibition of DNA repair proteins (including Rad51 and DNA-PK) in breast cancer cells (Figs. 2A, 2B&2C). We also evaluated γH2AX expression, which is a sensitive indicator of DNA DSB and corresponds to DSB repair in cells that are exposed to IR. The expression level of γH2AX was found to be significantly enhanced following the combined treatment compared with SAHA or IR alone *in vitro* and *in vivo* (Figs. 2B&4D). Moreover, the combination of IR with SAHA achieved radiosensitizing potential both in *in vitro* and in the orthotopic breast cancer mouse model (Figs. 1&4).

The article "Suberoylanilide Hydroxamic Acid, an Inhibitor of Histone Deacetylase, Enhances Radiosensitivity and Suppresses Lung Metastasis in Breast Cancer In Vitro and In Vivo" was published in 2013. Journal: PLoS One.

For most of the history of cancer therapy, apoptosis was thought to be the only mechanism of drug-induced cell death. More recently, it has been reported that a type II programmed cell death, autophagy, may participate in cancer therapy-induced cancer cell death [49]. However, a dual role for autophagy in cancer therapy has been reported both protecting against and promoting cell death [50]. Although substantial progress has been made in understanding the molecular control of autophagy and its regulation, a few studies answer questions that deal with the prediction of how and when the molecular machinery of autophagy affects cell death or cell survival [51]. Recent findings, including ours have demonstrated that activated autophagy is involved in chemo- and/or radiotherapy-induced cell killing [37], [38], [52]. Our current results also show that the combination of IR with SAHA induced remarkable autophagy but only minor apoptosis in 4T1 cells (Fig. 3). The induction of autophagy could be further demonstrated by our *in vivo* study of 4T1 orthotopic tumors, in which LC3 (a marker of autophagy) was increased following a combined treatment with SAHA and IR (Figs. 3D, 3E&4D). The combined treatment of 4T1 cells pre-treated with 3-MA, an inhibitor of autophagy, resulted in a significant reduction in cytotoxicity (Fig. 3G). In addition, although DNA damage plays an important role in the induction of autophagy [21], the exact mechanisms by which DNA damage triggers autophagy are unclear. Thus, more studies are needed to clarify the relationship between DNA damage and autophagy.

Recent evidence shows that one of the mechanisms whereby IR activates ER stress is the induction of DNA damage [26]. Thus, DSBs may serve as one link between IR and ER stress activation. Our results showed that IRE1α and the phosphorylation of eIF2α increased with the combined treatment, indicating that the combined treatment could induce ER stress in 4T1 cells (Fig. 2E). Similar to our finding, occurrence of ER stress has been reported to be associated with the induction of autophagy and upregulation of autophagic marker LC3 [53]. In mammalian cells, ER stress has been shown to facilitate the formation of autophagosomes, and induction of autophagy enables the removal of toxic misfolded proteins [54]. Healy et al. indicated that the growth arrest and DNA damage-inducible protein (GADD153) could serve as a main mediator of ER stress-induced cell death [55]. Therefore, DNA damage could induce ER stress and consequently autophagy. A better understanding of the signaling pathways controlling autophagy, DNA damage and ER stress will hopefully open new possibilities for the treatment of numerous cancers.

The article "Suberoylanilide Hydroxamic Acid, an Inhibitor of Histone Deacetylase, Enhances Radiosensitivity and Suppresses Lung Metastasis in Breast Cancer In Vitro and In Vivo" was published in 2013. Journal: PLoS One.

The majority of deaths in breast cancer patients are from metastases rather than primary tumors, and studies have shown that breast cancer preferentially metastasizes to the lung, liver, and bones. With up to 20% of these patients likely to develop metastatic disease, the identification and implementation of more effective therapies is a high priority [56]. In the present study, we demonstrated for the first time that SAHA significantly delayed lung metastases in an *in vivo* experimental metastasis animal model (Fig. 6). Our results showed that SAHA decreased lung weight and tumor volume compared to the control treatment (Figs. 6B&6C). Furthermore, a significant decrease in the number and size of tumors was observed in the lung sections from animals treated with SAHA (Fig. 6D). Mechanistically, our cellular data indicated that SAHA inhibited breast cancer cell migration through inhibiting the activity of MMP-9 (Figs. 5E&5F). MMPs have been implicated as possible mediators of invasion and metastasis in some cancers. Among the human MMPs, MMP-9 is the key enzyme that degrades type IV collagen. In addition, aberrant overexpression of MMP-9 has been found to be associated with an increased invasive potential in breast cancer cells [57]. Investigation into which additional metastasis-related proteins are involved in SAHA-induced migration inhibition is worth further analysis.

To our knowledge, this is the first report demonstrating that SAHA enhances the radiation response in a 4T1-luc orthotopic mouse model. In our animal model, SAHA plus IR showed better efficacy over individual treatments in delaying the growth of tumors. Furthermore, the combined treatment induced stronger cytotoxicity in breast cancer cells. One of the mechanisms whereby SAHA inhibited the cell’s capacity to repair IR-induced DNA damage by affecting the DNA repair pathways, could contribute to this combined effect. Induction of autophagy and ER stress could also be involved in the underlying mechanisms. In addition, we further found that SAHA inhibited the invasion and migration of breast cancer cells by inhibiting the activity of MMP-9 *in vitro*. Accordingly, in an *in vivo* experimental metastasis mouse model, SAHA significantly inhibited lung metastasis at non-cytotoxic concentrations. Based on these findings, we propose that SAHA could serve as a radiosensitizer or suppress lung metastasis by itself in breast cancer.
